The article "A novel necroptosis signature for predicting survival in lung adenocarcinoma" was retracted in 2024. Reasons: missing or withdrawn patient consent; concerns about the authorship.

# A novel necroptosis signature for predicting survival in lung adenocarcinoma

**DOI:** 10.1186/s12920-023-01748-9

**Published:** 2023-11-28

**Authors:** Kui Zang, Min Wang, Xingxing Zhu, Bin Yao, Ying Huang

**Affiliations:** Department of ICU, the Affiliated Huaian No.1 People’s Hospital of Nanjing Medical University, Jiangsu Province, Huai’an, No.1, Huanghe West Road, Huaiyin District 223300 China

**Keywords:** Necroptosis, Signature, Prognosis, Prediction, Immune checkpoint, LUAD

## Abstract

**Background:**

To explore the necroptosis-related genes (NRGs) signature and its predictive values in lung adenocarcinoma (LUAD).

**Methods:**

The training cohort consisted of tumor samples from The Cancer Genome Atlas, and the validation set comprised data from the Gene Expression Omnibus. Univariate and multivariate Cox regression analyses were applied to identify the prognostic NRG signature as an independent molecular indicator. Correlation analysis was used for the association assessment between the NRG signature and immune checkpoint molecules.

**Results:**

NRGs involved in necroptosis and immune NOD-like receptor signaling. The NRG signature based on eight NRGs can divide tumors into high-risk and low-risk groups, which was significantly associated with worse survival. Multivariate Cox regression analysis showed that this NRG signature remained an independent prognostic indicator. Stratification analyses demonstrated that this NRG signature was still effective for predicting survival in each stratum of age, gender, and tumor stage. The ROC curve showed a good predictive ability using the NRG signature in the validation cohort (AUC = 0.81). The NRG signature was related to immune checkpoint molecules PD − 1, PD-L1, and PD-L2.

**Conclusions:**

The NRG signature could be a novel predictor of the prognosis and may become a potential therapeutic target in LUAD.

**Supplementary Information:**

The online version contains supplementary material available at 10.1186/s12920-023-01748-9.

## Background

Lung cancer is the second most common human malignancy and the highest cause of cancer-related deaths in the world [1]. The global cancer statistics show an estimated 2.2 million new cancer cases and 1.8 million deaths [1]. Non-small cell lung cancer (NSCLC) is the most commonly diagnosed lung cancer type. Although surgery, chemotherapy, radiotherapy, targeted therapy, and immunotherapy demonstrate numerous advances in treating NSCLC. The 5-year survival rate remains depressing [2, 3]. Lung adenocarcinoma (LUAD) and squamous cell carcinoma (LUSC) are the most common NSCLC subtypes. LUAD and LUSC show significantly distinct at the transcriptomic level and cellular control networks [4]. LUAD accounts for approximately 40% of lung cancer cases and is the most common type [4].

The article "A novel necroptosis signature for predicting survival in lung adenocarcinoma" was retracted in 2024. Reasons: missing or withdrawn patient consent; concerns about the authorship.

Necroptosis is a regulated necrotic cell death that is distinguished from classical caspase-dependent apoptosis. It is mainly mediated by receptor-interacting protein kinase 1 (RIPK1) and RIPK3, and mixed lineage kinase domain-like (MLKL) [5]. Accumulating evidence demonstrates that necroptosis plays a vital role in regulating multiple physiological and pathological functions such as cell survival, cell proliferation, the production of pro-inflammatory cytokines, the release of damage-associated molecule patterns (DAMPs), inflammation, and angiogenesis [5–7]. Necroptosis has a prominent role in tumorigenesis, tumor progression, cancer metastasis and prognosis, and immune regulation [8, 9]. Necroptosis may contribute to the augmented therapeutic efficiency of tumors by accelerating cancer cell death or enhancing the sensitivity of tumor cells [10, 11]. Some studies have reported the necroptosis-related gene (NRG) signature can predict poor prognosis in some human cancers, including NSCLC [12–14]. However, little analysis was conducted on the role between the NRG signature and LUAD. We studied the interaction of the NRG signature with prognosis, clinical molecular characteristics, and immune checkpoint molecules in LUAD.

The current study established a prognostic score model according to the NRGs. Next, we investigated the molecular signature with the prognostic and predictive efficacy and validated this molecular signature for the stratification of LUAD. Our study will provide reliable evidence for treatment optimization and further clarification of individual patients with LUAD.

## Methods

### Data processing and clinical data

We obtained transcriptomic expression data and clinicopathological information of LUAD patients from The Cancer Genome Atlas-Sarcoma (TCGA-LUAD) cohort. The RNA-seq data were normalized using the Trimmed Mean of M-values (TMM) method. Gene expression profiles were log2 transformed values [log2(x + 1)]. Patients with incomplete clinical survival data were excluded. Finally, 494 LUAD cases with sufficient survival data were enrolled as a training cohort. In addition, we acquired data from the Gene Expression Omnibus (GEO) for a substantial cohort of LUAD tumor patients (GSE72094). This dataset was subjected to IRON normalization and underwent a log2 transformation. Forty-four patients with incomplete survival data were excluded. The data set GSE72094 was used as a verification cohort, including 398 cases with clinical prognostic information. The clinicopathological characteristics from the training and validation cohorts are presented in Table S1.

The article "A novel necroptosis signature for predicting survival in lung adenocarcinoma" was retracted in 2024. Reasons: missing or withdrawn patient consent; concerns about the authorship.

### Identification of NRGs and functional analysis

We acquired necroptosis-related genes (NRGs) from the GSEA (M24779.gmt), KEGG pathway (hsa04217), and previous studies [15, 16]. We ultimately identified 204 NRGs in the present study (Table S2). The functional enrichment analysis was further analyzed with Metascape. Metascape provides a comprehensive gene list annotation and analysis resource for experimental biologists, including functional enrichment analysis [17].

### Construction of the NRG signature

Based on 204 NRGs obtained, we constructed a novel NRG signature using the following process. First, a univariate Cox regression analysis was carried out to determine the NRGs associated with overall survival. *P* values with < 0.05 for these prognostic genes were included. The final 35 significant prognostic genes were found in the training set. Second, to obtain the final necroptosis-related prognostic genes, multivariate Cox regression analysis with the two-step method was employed to filter features to establish a risk model. Finally, 8 NRGs were identified in our study. The following formula was used to calculate the NRGscore for each tumor sample: Σ^n^_i=1_ expression_i_ ∗ corresponding coefficient_i_.

### The NRG signature for predicting immune checkpoint molecules

Immune checkpoint blockade (ICB) therapy [immune-checkpoint proteins programmed cell death 1 (PD-1) and its ligands (PD-L1 and PD-L2) and cytotoxic T-lymphocyte-associated protein 4 (CTLA-4) targets] has revolutionized the treatment of human cancers, including lung cancer. However, only a subset of patients achieves optimal clinical outcomes from ICB therapy [18, 19]. We explored whether the NRG signature could be a potential predictor of ICB molecules.

### Statistical analysis

Spearman’s correlation test was performed to evaluate the association between NRGscore and immune checkpoint molecules. The association between the NRG signature and different clinical and mutational features was assessed utilizing the Wilcoxon test. The median value of the training set was determined to find the cut-off value. LUAD cases were divided into high and low-risk score groups. Kaplan–Meier(K-M) analysis with the log-rank test was conducted to compare the survival differences between the low-risk and high-risk groups. The “timeROC” package created a time-dependent receiver-operating characteristic (ROC) curve to evaluate the predictive ability of the NRG signature. The prognostic risk [(hazard ratio, HR with a 95% confidence interval (CI)] was calculated for the NRG signature using a Cox proportional hazard model. Univariate and multivariate Cox analyses were performed to determine whether the NRG signature can be an independent prognostic factor in LUAD, along with the clinicopathological variables in the training and verification cohorts. Stratification analyses were conducted based on clinicopathological variables such as age, gender, tumor stage, KRAS mutation, TP53 mutation, and EGFR mutation status. All analyses were performed by using R software (version 3.6.3; R Foundation for Statistical Computing, Vienna, Austria).

The article "A novel necroptosis signature for predicting survival in lung adenocarcinoma" was retracted in 2024. Reasons: missing or withdrawn patient consent; concerns about the authorship.

## Results

### Development of the NRG signature

NRGs were conducted for functional enrichment analysis. Metascape analysis demonstrated that these NRGs were most closely enriched in necroptosis. The biological functions and pathways also showed that the NOD-like receptor signaling, programmed necrotic cell death, neutrophil extracellular trap formation, death receptor signaling, apoptosis, and regulated necrosis were linked with NRGs (Fig. 1A).

**Fig. 1:** Construction of the NRG signature. (**A**) Functional enrichment analysis of NRGs with Metascape. (**B**) Using multivariate Cox regression analysis, a forest plot showing the final eight NRGs in the NRG signature

A multivariate Cox regression model was applied to select the final NRGs in the training set. Ultimately, eight NRGs were used to establish a novel model in LUAD (Fig. 1B). The prognostic index was performed according to the expression levels of the genes and their corresponding coefficients. The formula used to calculate risk scores was as follows: (0.18 × ID1 expression) + (-0.35 × SIRT2 expression) + (0.307 × PPIA expression) + (0.238 × PYGB expression) + (0.276 × TICAM2 expression) + (-0.106 × ALK expression) + (-0.158 × IL33 expression) + (0.20 × BIRC3 expression).

### The NRG signature predicts survival in LUAD

To understand the prognostic potential of the NRG signature, we investigated its capability to predict survival outcomes in patients with LUAD. Figure 2 A demonstrates tumor samples’ distribution and survival status for the NRG signature in the training and validation cohorts, suggesting that a higher NRG score had shorter survival. Kaplan–Meier survival curves revealed that LUAD patients in the high NRG score group had a significantly poorer prognosis than cases with LUAD in the low NRG score group (*P* < 0.001) (Fig. 2B). The time-dependent ROC curves were performed to assess the predictive performance of the NRG signature. The areas under the curve (AUC) value for five years was 0.81 in the validation cohort (Fig. 2C), indicating the NRG signature’s advantage as a robust tool for survival prediction. Moreover, by utilizing the designated cut-off value as a threshold, we observed consistent performance metrics (sensitivity, specificity, positive predictive value [PPV], negative predictive value [NPV], and accuracy) in both the training and validation cohorts.

The article "A novel necroptosis signature for predicting survival in lung adenocarcinoma" was retracted in 2024. Reasons: missing or withdrawn patient consent; concerns about the authorship.

**Fig. 2:** The NRG signature for predicting survival in the training and validation cohorts of LUAD. (**A**) The distribution and survival status of tumors with LUAD for the NRG signature. (**B**) Kaplan–Meier survival curves between the high-risk and low-risk groups (*P* < 0.001). (**C**) Time-dependent ROC analyses at 1, 3, and 5 years in the training set (sensitivity = 0.62, specificity = 0.56, positive predictive value (PPV) = 0.4, negative predictive value (NPV) = 0.75, and accuracy = 0.58) and the validation set (sensitivity = 0.63, specificity = 0.56, PPV = 0.36, NPV = 0.79, and accuracy = 0.58)

### Independent prognostic value of the NRG signature

We evaluated the independence of the NRG signature by univariate and multivariate Cox regression analyses in the training and validation sets. Univariate Cox analysis demonstrated that the high NRG score group was significantly correlated with worse prognosis in LUAD (training cohort: HR = 2.480, 95% CI = 1.798–3.419, *P* < 0.001; validation cohort: HR = 2.003, 95% CI = 1.367–2.935, *P* < 0.001). The NRG signature consistently emerged as an independent prognostic predictor in subsequent multivariate Cox regression analyses. This was evident even after adjusting for clinical features such as tumor stage, T, M, and N classifications in the training cohort (HR = 2.074, 95% CI = 1.400-3.073, *P* < 0.001). Similarly, when adjustments were made for gender, tumor stage, KRAS mutation, and EGFR mutation in the validation cohort, the results of the NRG signature remained significant (HR = 2.026, 95% CI = 1.371–2.993, *P* < 0.001) (Table 1).

**Table 1:** Univariate and multivariate Cox analyses of the NRG signature

Variables	Univariate Cox analysis		Multivariate Cox analysis	
	HR (95% CI)	*P*	HR (95% CI)	*P*
Training cohort				
NRG signature (high vs. low)	2.480 (1.798–3.419)	< 0.001	2.074 (1.400-3.073)	< 0.001
Age (≥ 65 vs. < 65 years)	1.210 (0.883–1.657)	0.235		
Gender (male vs. female)	1.047 (0.768–1.426)	0.773		
Tumor stage (stage 3–4 vs. 1–2)	2.805 (2.027–3.882)	< 0.001	1.774 (1.039–3.029)	0.036
Smoking (yes vs. no)	0.894 (0.568–1.406)	0.627		
T (T 3–4 vs. 1–2)	2.405 (1.606–3.603)	< 0.001	1.438 (0.865–2.390)	0.161
M (positive vs. negative)	1.857 (1.062–3.247)	0.03	1.031 (0.524–2.029)	0.929
N (positive vs. negative)	2.642 (1.930–3.618)	< 0.001	1.771 (1.137–2.758)	0.011
Validation cohort				
NRG signature (high vs. low)	2.003 (1.367–2.935)	< 0.001	2.026 (1.371–2.993)	< 0.001
Age (≥ 65 vs. < 65 years)	1.379 (0.889–2.137)	0.151		
Gender (male vs. female)	1.552 (1.072–2.246)	0.020	1.521 (1.039–2.226)	0.031
Tumor stage (stage 3–4 vs. 1–2)	2.607 (1.736–3.914)	< 0.001	2.881 (1.905–4.358)	< 0.001
Smoking (yes vs. no)	1.369 (0.597–3.139)	0.459		
KRAS mutation (positive vs. negative)	1.456 (1.001–2.118)	0.049	1.249 (0.851–1.833)	0.256
EGFR mutation (positive vs. negative)	0.262 (0.096–0.710)	0.008	0.340 (0.123–0.938)	0.037
TP53 mutation (positive vs. negative)	1.235 (0.820–1.860)	0.313		

h: hazard ratio; CI: confidence interval

The article "A novel necroptosis signature for predicting survival in lung adenocarcinoma" was retracted in 2024. Reasons: missing or withdrawn patient consent; concerns about the authorship.

### Predictive performance of the NRG signature in various clinical and mutational variables

According to age (≥ 65 vs. < 65 years), gender (male and female), tumor stage (stage 3–4: advanced-stage and stage 1–2: early-stage), KRAS mutation status (positive and negative), TP53 mutation status (positive and negative), and EGFR mutation status (positive and negative) in the entire data (Figs. 3 and 4), we performed stratification analyses. Figure 3 shows a stratification analysis of age, gender, and tumor stage. We found that the high-risk group had a worse survival than the low-risk group in each stratum of age, gender, and tumor stage (all *P* values < 0.01). This suggested that our NRG signature was still an effective indicator for predicting prognosis in older or younger, male or female, and advanced-stage or early-stage patients with LUAD. The NRG signature in various mutational characteristics demonstrated that the high-risk group had poor prognosis than the low-risk group in patients with KRAS wild − type (negative), EGFR wild − type, and TP53 wild-type (all *P* values < 0.01), which indicated that this signature could be an effective tool for survival prediction in LUAD with wild − type KRAS, EGFR, or TP53.

**Fig. 3:** Kaplan-Meier results of the NRG signature using stratification analyses of age, gender, and tumor stage, including (**A**) ≥ 65 years, (**B**) < 65 years, (**C**) male, (**D**) female, (E) stage 3 − 4, and (F) stage 1 − 2

**Fig. 4:** Kaplan-Meier results of the NRG signature using stratification analyses of KRAS mutation status, TP53 mutation status, and EGFR mutation status, including (**A**) KRAS mutation, (**B**) KRAS wild − type (negative), (**C**) EGFR mutation, (**D**) EGFR wild − type (negative), (**E**)TP53 mutation, (**F**) TP53 wild − type (negative)

We evaluated the correlation between the NRG signature and various clinical features, such as age, gender, tumor stage, T classification, lymph node status, and distal metastasis (Fig. 5A-F). In addition, we investigated the association of the NRG signature with mutational features, such as EGFR mutation, KRAS mutation, and TP53 mutation status (Fig. 5G-I). The results indicated significant correlations between the NRG signature and various factors: gender (*P* = 0.01), tumor stage (*P* = 0.012), T classification (*P* = 0.003), lymph node metastasis status (*P* < 0.001), KRAS mutation status (*P* = 0.02), and TP53 mutation status (*P* < 0.001). Specifically, higher NRG signature scores were observed in male patients, those with advanced tumor stages, those classified as T 3–4, individuals presenting with lymph node metastasis, and patients carrying KRAS or TP53 mutations.

The article "A novel necroptosis signature for predicting survival in lung adenocarcinoma" was retracted in 2024. Reasons: missing or withdrawn patient consent; concerns about the authorship.

**Fig. 5:** Association between the NRG signature and various clinical features (**A-F**) and mutational features (**G-I**)

### The NRG signature for predicting immune checkpoint molecules

We investigated whether the NRG signature could predict immune checkpoint molecules. We examined the relationship between the NRG signature and the immune checkpoint molecules such as PD-1 and its ligands PD-L1, PD-L2, and CTLA-4 in LUAD (Figure S1). The results demonstrated that our signature was positively correlated with the expression levels of genes encoding the immune checkpoint proteins: PD-1 (PDCD1) (r = 0.12, *P* = 0.010), PD-L1 (CD274) (r = 0.15, *P* = 0.001), and PD-L2 (PDCD1LG2) (r = 0.15, *P* = 0.001).

### Investigation of non-necroptosis genes as a control signature

We selected control signatures consisting of non-necroptosis genes to identify any possible spurious associations. Metascape analysis revealed functional enrichment results indicating a strong correlation between non-necroptosis genes and processes such as cell cycle and DNA replication (Fig. 6A). According to the results of univariate Cox regression analysis, lasso regression analysis, and the multivariate Cox regression model, we developed a non-NRG signature comprising ten non-necroptosis genes (Figure S2A).

**Fig. 6:** Construction of the non-NRG signature. (**A**) Functional enrichment analysis from Metascape analysis for the selected non-necroptosis genes using univariate Cox regression analysis with a significance level of *P* < 0.01. (**B**) Time-dependent ROC analyses at 5 years in the validation cohort (NRG signature: AUC = 0.81; non-NRG signature: AUC = 0.66)

Kaplan–Meier survival analyses were conducted to examine the prognostic implications of the non-NRG signature in LUAD. The results revealed a significant association between the non-NRG signature and an unfavorable prognosis (*P* < 0.05) (Figure S2B). The time-dependent ROC curves demonstrated a low AUC value (AUC = 0.66) for the non-NRG signature at 5 years in the validation set (Fig. 6B and Figure S2C).

The non-NRG signature was further evaluated in association with various clinical features, mutational features, and immune checkpoint molecules. The non-NRG signature exhibited significant correlations (*P* < 0.05) with several clinical features, including gender, tumor stage, T classification, lymph node metastasis, and distal metastasis, as well as mutational features such as EGFR mutation, KRAS mutation, and TP53 mutation (Figure S3). The analysis of the non-NRG signature in relation to immune checkpoint molecules revealed a significant positive correlation with only PD-L1 and PD-L2 (*P* < 0.05) (Figure S4).

The article "A novel necroptosis signature for predicting survival in lung adenocarcinoma" was retracted in 2024. Reasons: missing or withdrawn patient consent; concerns about the authorship.

## Discussion

LUAD is the largest lung cancer subtype, and it is more common in women and nonsmokers. There appears to be a clear distinction between LUAD and LUSC in terms of molecular profiles and driver genetic alterations. For example, a driving p53/p63/p73 axis is significantly correlated with LUSC but not with LUAD. EGFR mutations, receptor tyrosine kinases mutations, and EML4-ALK rearrangements were more frequent in LUAD but rare in LUSC [4, 20, 21]. These can result in diversities in therapeutic options. Studies have reported that a reliable prognostic biomarker should predict prognosis, cancer classification, and therapy response, which can be utilized to standardize the evaluation of personalized therapies. [22, 23], but their accuracy of survival prediction and response to treatment remains limited. Here, we integrated multiple prognostic biomarkers-based risk group stratification to further improve the optimal selection for predicting survival and therapy in LUAD. In the current work, we developed and validated a novel NRG signature for survival prediction in patients with LUAD.

We firstly screened out 204 NRGs and finally identified 8 NRGs with significant prognostic values in our molecular signature. We constructed a prognostic index according to the final eight NRGs and found that tumors with LUAD could be classified into two risk groups between which the survival differed significantly. Our NRG signature was closely associated with worse prognosis and could be an independent prognostic factor for LUAD. This NRG signature was also correlated with immune checkpoint molecules PD-1, PD-L1, and PD-L2. In addition, we selected non-necroptosis genes as control signatures. We developed a non-NRG signature and found that the NRG signature achieved a significantly higher AUC value (0.81) compared to the non-NRG signature (AUC = 0.66). The functional enrichment analysis highlighted a pronounced association of NRGs with necroptosis. In contrast, non-necroptosis genes were significantly linked to the cell cycle.

Our molecular signature consisted of eight NRGs. Among them, ID1 is related to epithelial-mesenchymal transition (EMT)-related proteins and some signaling pathways such as the WNT pathway and TGF-β signaling. ID1 plays a facilitating role in tumorous angiogenesis, cancer metastasis, and drug resistance [24]. ID1 enhances chemotherapy sensitivity and induces necroptosis by activating RIP1/RIP3/MLKL pathway in NSCLC [25]. SIRT2 inhibits T-cell metabolism [26], and it has a key role in cell proliferation, migration and invasion, metabolism, stem cell-like features, and autophagy [27]. SIRT2 expression is closely associated with prognosis in patients with LUAD but not LUSC [28]. PPIA expression is found to be correlated with poor survival in many cancers, including LUAD [29]. PPIA may serve as a potential new target for resistant multiple myeloma [30]. PYGB contributes to cell proliferation, migration, and invasion via activating the Wnt signaling pathway and is related to poor prognosis in NSCLC [31]. ALK is involved in the initiation and progression of various cancers and its overexpression has been reported in cancer [32]. ALK overexpression is associated with worse prognosis, and ALK downregulation suppresses cell viability and induces cell death in LUAD [33]. IL33 release is a marker for response to necroptosis [34]. IL33 induces T cell proliferation and IL-17 secretion, thereby promoting antitumor effects in LUAD. IL33 expression is related to favorable survival in patients with LUAD [35]. BIRC3 mutation is associated with worse prognosis in chronic lymphocytic leukemia [36]. BIRC3 expression is observed in human NSCLC [37]. In addition, the NRG signature is reported to be associated with worse prognosis in several human cancers, including NSCLC [12–14]. Our results were consistent with these previous studies, and we found that our NRG signature is closely related to poor prognosis and could stratify patients into the high-risk and low-risk group in LUAD. Then, multivariate Cox analysis suggested that this NRG signature remained an independent molecular indicator for predicting survival in LUAD. We further investigated the predictive value of the NRG signature in various clinical and molecular characteristics. We observed that our signature remained a powerful tool for survival prediction in older or younger, male or female, early-stage or advanced-stage, KRAS negative, EGFR negative, or TP53 negative patients with LUAD. These analyses proved that this NRG signature was a strongly effective and good performance for survival prediction in LUAD.

The article "A novel necroptosis signature for predicting survival in lung adenocarcinoma" was retracted in 2024. Reasons: missing or withdrawn patient consent; concerns about the authorship.

ICB with PD-1/PD-L1 antibodies has revolutionized the therapy of several cancers, such as NSCLC (LUAD and LUSC). However, ICB has limited success in LUAD. LUAD generally has lower TMB, lower prevalence of PD-L1 expression, more uninflamed and immunosuppressive TME, and high prevalence of active driver mutations (EGFR mutation) than LUSC [4, 38]. These reasons can explain the poorer results and less benefits of ICB immunotherapy in LUAD in part. We found that our signature was associated with ICB molecules (PD-1, PD-L1, and PD-L2), which suggests that our NRG signature may predict immune checkpoint molecules in LUAD. To enhance the clinical relevance, further study is necessary to evaluate the correlation between the NRG signature and the expression of immunohistochemistry (IHC) proteins of immune checkpoints using stained slides in the future.

## Conclusion

In conclusion, we established a valuable NRG signature, which may effectively predict survival of patients with LUAD. Our findings provided new evidence for individualized therapy for therapeutic decisions. Further research for elucidating the value of the NRG signature in LUAD is in need.

### Electronic supplementary material

Below is the link to the electronic supplementary material.

Supplementary Material 1

Supplementary Material 2

Supplementary Material 3

## Data Availability

The datasets analyzed during the current study are available in the GEO repository, (https://www.ncbi.nlm.nih.gov/geo, accession number GSE72094).
